This article has been retracted.

# The Influence of PDCA Cycle Management Mode on the Enthusiasm, Efficiency, and Teamwork Ability of Nurses

**DOI:** 10.1155/2022/9352735

**Published:** 2022-07-08

**Authors:** Na Pan, Yu Ye Luo, Qiu Xia Duan

**Affiliations:** ^1^Obstetrics Department, Taikang Tongji (Wuhan) Hospital, Wuhan City, Hubei Province 430050, China; ^2^Nursing Department of Taikang Tongji (Wuhan) Hospital, Wuhan City, Hubei Province 430050, China; ^3^Thoracic Heart and Urology Department of Taikang Tongji (Wuhan) Hospital, Wuhan City, Hubei Province 430050, China

## Abstract

**Background:**

The PDCA cycle consists of four stages: P (plan), D (design), C (check), and A (action). With the wide acceptance of PDCA cycle, there is an urgent need to verify the effect of combining this concept with clinical nursing work. Therefore, on the basis of in-depth study of a large number of related literature, the influence of PDCA cycle management mode on nurses' work efficiency, work enthusiasm, and teamwork ability was explored, so as to provide reference experience for exploring the nursing quality management model adapted to the development of medicine.

**Objective:**

To explore the application of PDCA circulation management mode in clinical nursing work and to explore its influence on the work efficiency, enthusiasm, and team cooperation ability of nurses.

**Methods:**

From January 2019 to January 2021, the patients were divided into two groups. The control group received routine nursing care, and the research group received the PDCA circulation management mode. Both groups of nurses received one-year training. The nursing quality, the ability of teamwork, the scores of personal quality control in clinical departments, the scores of nursing satisfaction, the number of problems in nursing document quality management, and nurses' enthusiasm were compared between the two groups.

**Results:**

The scores of relationships and family and work balance were greater than those of the control group. The nursing quality result suggested the nursing quality of gynecological operation area, emergency operation area, comprehensive operation area, and surgical operation area in research nurses was significantly better than the control cases (*P* < 0.05). The quality management of nursing documents showed that the number of problems in nursing documents such as nursing record displayed fewer than control group (*P* < 0.05). The personal quality-controlled checking in medical department showed that the points of ward governance, head nurse management quality control examination, first-level nursing, recovery, publications on therapeutics, pill governance, and healthcare documentation in the research group were higher than control group (*P* < 0.05). The teamwork ability implied the scores of interpersonal communications, problem definition, project division, team evaluation assistance and motivation, data collection, interpretation, and extraction of results in the observation group were remarkably greater than those of control group (*P* < 0.05). The satisfaction mark showed that the scores of care information exchange, advanced technologies, attitude towards care providing, healthcare establishing, knowledge publicity, and learning in the researches were markedly more than those of the control group (*P* < 0.05).

**Conclusion:**

Compared with the traditional clinical nursing management, the use of the PDCA circulation management mode can effectively improve the quality of hospital nursing work, strengthen nurses' ability of teamwork, improve nurses' work efficiency and enthusiasm, enhance their sense of achievement of clinical nursing work, then improve patient satisfaction, and enhance the reputation and competitiveness of hospitals. Therefore, the PDCA management model is worth popularizing and applying in clinic.

## 1. Introduction

In the overall medical work of the hospital, nursing work is an important part of clinical service, so the quality of nursing can reflect the quality of hospital management and medical level, which is directly related to the reputation of the hospital and the life and health of nurses [1]; thus, it can be seen as a vital marker improving the quality of hospital nursing. Although both the medical structure and the patient group have positive and urgent requirements for improving nursing treatment, there are still some problems in the actual nursing work, such as service concept, personnel quality, and management methods, which hinder the further improvement of nursing quality [2]. The PDCA cycle, also known as the “Deming Ring,” consists of four stages: P (plan), plan; D (design), design; C (check), inspection; and A (action), processing. After years of wide application in various important fields, it is generally regarded as a kind of step-by-step management work. Numerous registered-nurse scholars have successfully made contributions to the administration of high-quality care [3]. To implement and run the PDCA theory standardization process, the key lies in the whole process management, the overall mobilization for all staff, and a comprehensive grasp of the actual situation of each participant [4]. It has been demonstrated the application of PDCA principle in patient care can implement the requirements of nursing management, enrich the connotation of nursing service, improve the psychological construction of nurses, and improve the nursing quality steadily [5, 6]. With the acceptance widely of PDCA cycle, there is an urgent need for empirical research with nurses as the main body to further verify the effect of the combination of this concept and clinical nursing work. Therefore, on the basis of in-depth study of a large number of related literatures, our investigation explored the impact of the PDCA cycle management model on the work efficiency, enthusiasm, and team cooperation ability of nurses, so as to provide reference experience for seeking a nursing quality management model adapted to the development of medicine.

## 2. Materials and Methods

### 2.1. General Information

There were two groups from Jan. 2019 to Jan. 2021 in this investigation. The control nurses accepted the conventional care, and the research group accepted the PDCA cycle management model. Both nurses were cared for a period of one year. 80 nurses were selected in the corresponding year. The control's nurses conducted conventional care, while the experimental nurses carried out the PDCA circulation care mode.

The research nursing team comprised of 2 male nurses and 78 female nurses. These nurses ranged in age from 20 to 53 years old, with just an overall mean of 31.64 ± 1.33. The investigation nurses' age ranged from 13 to 83 years old with an overall mean of 45.64 ± 3.64. The control team comprised of 1 male and 79 female nurses. Their age was 20 to 52 years old with overall mean of 31.56 ± 1.34 years old. The control cases' ages were 13 to 83 years old with mean of 45.13 ± 3.55 years. There was no significant difference in age and gender between the two groups (*P* > 0.05).

### 2.2. Methods

The control group needs to accept the routine nursing management in the ward in accordance with the requirements of the routine management of the hospital. Under the above premise, the research group will also use the PDCA cycle management model. The study is divided into four stages, as follows.

#### 2.2.1. Planning Stage

Under the direction of the clinic's commission (the quality management committee refers to the director of the clinical work of the hospital as the director of the committee, and the director of the nursing department of the hospital as the deputy director; other members are composed of heads of other relevant departments. And select a suitable person to serve as the secretary of the committee) a multilevel personnel structure was established composed of quality management leadership team, quality control person in charge, head nurses in each ward, and all nurses in each ward. Among them, the person in charge of the accusation will be the director, and the team will be made up of the heads of each ward's nurses. The content of quality control requires the five aspects: special care governance, ward care, rescue and treatment materials management, head nurse governance, and nursing document management. At the same time, we plan to carry out nursing quality competition in the hospital and formulate a staff training plan for the relevant management content, in order to introduce the competitive mechanism, promote the formation of a virtuous circle of assessment, and improve the ability of all personnel.

#### 2.2.2. Implementation Stage

The persons in charge and their members should conduct extensive research on the definition and the quality standard and conduct regular assessment. The head nurses in each ward need to raise questions according to the characteristics of their departments and the difficulties and deficiencies encountered in their work, put forward rectification suggestions item by item according to the relevant contents of the quality standards, and organize all personnel to participate in the formulation of the implementation plan. The final plan can be implemented in the ward after evaluation and approval by the nursing department. The quality assurance guiding individuals involved are regularly organized by the guiding team to know relevant expertise, and each member needs to write an article based on their own work experience. At the implementation level, the circular management mode is adopted in the whole implementation process; the details are as follows: the leading group needs to implement the management responsibilities of five projects, namely, aid and therapy information administration, ward management, exceptional first-level of primary care, head nurse, and nursing document administration to the responsible persons; the person in charge shall inspect each ward according to the specific conditions and adjust the content in time according to the implementation situation. The head nurse of each ward shall carry out his duties according to the management plan from the above five aspects to the person responsible for quality control and supervision in Kone, and the responsible person shall supervise and guide the clinical work; among them, the leading group needs to organize hospital-scale education and evaluation regularly and formulate strict standards. The head nurses in each ward should organize regular meetings, refine the criteria for achieving quality and evaluation approaches according to the characteristics of the ward, analyze the problems found in the inspection, formulate a reasonable rectification plan, and urge all departments to set up internal quality control teams to form a good atmosphere of full staff participation, full staff supervision, their responsibilities, cooperation, and mutual assistance; all clinical nurses should be familiar with and master the aforementioned duties and tasks and strictly carry out them.

#### 2.2.3. Inspection Stage

A perfect and effective inspection system composed of personal self-examination, ward inspection, quality control person-in-charge inspection, and phased inspection according to key points was established. First of all, healthcare workers should self-assess their regular assigned tasks and division of tasks in light of the level of care judging criteria, recording them in a standardized manner. The head nurse should carry out a comprehensive examination and standard record one time per week depending on the nursing quality evaluation standard, summarize it regularly, and report it to the nursing department. The person in charge of the accusation is to conduct a comprehensive inspection of all clinical departments of the hospital every three months, and the key departments are adjusted once a month, concentrating on the performance improvement points identified within every bureau's rectifying strategy.

#### 2.2.4. Summary and Treatment Stage

Each clinical nurse reports the self-check situation during the shift change; the nurse manager presents an analysis of the findings and discusses them at a technical seminar, which is helpful to revise the rectification objectives and improvement measures in time. The quality evaluation results of the participating employees determine their performance bonuses. The examination results of the person in charge are reported at the clinical quality governance board and feedback to the hospital information system, focusing on the analysis of universal or stubborn problems, the recommended timely feedback improved the measures and proposals related to medical units, and the achievements and experiences gained should be shared in time and maintained continuously and effectively. For the emerging problems, we need to revise the management standards, combined with experience to promote the next PDCA cycle.

### 2.3. Observation Index

#### 2.3.1. Enthusiasm for Work

In nurses' work enthusiasm [7], the work enthusiasm of the two groups of nurses was evaluated by the job satisfaction rating scale, which included 38 items. There are 8 dimensions, including work itself, workload, personal growth and development, job recognition, work management, relationship with colleagues, and family and work balance. Each item can obtain 1-5 score(s), and the overall points are 38-190. The Cronbach's table is *α* = 0.94.

#### 2.3.2. Nursing Quality in each District

In work quality-related indicators [8], the performance distribution management model was carried out in gynecological operation area, comprehensive operation area, emergency operation area, and surgical operation area, and the nursing quality in the first and last two periods was evaluated. The nursing department assessed the nursing quality in four areas of specialist quality twice a month. The quality-of-care accounting point was carried out based on 30% specialist quality, 40% nursing safety, and 30% nursing norms, with a total score of 100 points.

#### 2.3.3. The Number of Issues with Healthcare File Quality Control

Statistics were compiled on the series of issues that existed in the quality control of healthcare files in the two different groups, which included temperature sheets, physician's orders, assessment sheets, and nursing records.

#### 2.3.4. Personal Quality Check Investigation Score in Medical Office

The assessment criteria of healthcare control in clinical units of the hospital were used as the evaluation index [9–11]. The principle categorizes patient care quality control into 5 factors. Ward management focuses on nurses' mastery of basic medical knowledge; care file administration focuses on whether nursing staff can track nursing processes in accordance with rules and codes; and nursing supervisor governance focuses on complete and accurate guidance. The quality assurance criterion of recovery and therapies publications/medicine primarily examines whether the equipment and prescription pills are managed in the hospital, whereas the special first-level nursing interventions primarily considers whether nursing staff could provide timely, reliable, and successful nursing for critically ill patients.

#### 2.3.5. Teamwork Ability [12]

The evaluation of teamwork ability will be scored by a number of judges from different specialties and different wards, and the scoring criteria use the dimensional scoring method including data collection, interpretation of information, extraction of results, interpersonal communication, team evaluation assistance and motivation, problem definition, and project division of labor.

#### 2.3.6. The Satisfied Marks

In the evaluation of nurses' satisfaction [13], the questionnaire survey was performed. The survey form had ten items and dependent variables (care information exchange, advanced technologies, attitude towards care providing, healthcare establishing, knowledge publicity, and learning). Each question was worth of 1-20 points with a total of 20-100 points. The higher the score, the higher the patient satisfaction.

### 2.4. Statistical Analysis

Using the SPSS 24.0 software, the data were calculated and expressed as *x̅*±*s*. Two different groups were taken comparison by the *t* test, and *n* (%) was analyzed and represented the counting data. The distinction was clinically meaningful (*P* < 0.05).

## 3. Results

### 3.1. Comparison of Work Enthusiasm

The results of work enthusiasm showed that the work itself, workload, personal growth and development, job recognition, work management, relationship with colleagues, and family and work balance were higher than those in the control group, and the difference was statistically significant (*P* < 0.05) (see Table 1).

### 3.2. Comparison of Nursing Quality in each Area

The performance distribution management model was carried out in the gynecological operation area, comprehensive operation area, emergency operation area, and surgical operation area, and the nursing quality in the first and last two periods was evaluated. The nursing quality data of each area showed that the nursing quality of the gynecological operation area, comprehensive operation area, emergency operation area, and surgical operation area of the research group was higher than that of the control group, and the difference was statistically significant (*P* < 0.05) (see Figure 1).

### 3.3. Comparison of the Number of Problems in the Quality Management of Nursing Documents

The data of problems in the quality management of nursing documents showed that the number of problems in body temperature sheet, doctor's order, evaluation form, nursing record sheet, and other document in the research group was significantly lower than that in the control group (*P* < 0.05) (see Figure 2).

### 3.4. Comparison of Individual Quality Control Examination Scores in Clinical Departments

The results of single quality control inspection of clinical departments found that the scores of ward management, head nurse management quality control inspection, intensive care first-level nursing, rescue, treatment items, drug management, nursing documents, etc. in the research group were higher than those in the control group, and the difference was statistically significant (*P* < 0.05) (see Table 2).

### 3.5. Comparison of Teamwork Ability

The data of teamwork ability showed that interpersonal communication, team evaluation assistance, motivation, problem definition, interpretation of information, score of extraction results, project division of labor, and data collection in the research group were significantly higher than those in the control group (*P* < 0.05) (see Table 3).

### 3.6. Comparison of Satisfaction Score

The satisfaction score data showed that the scores of nursing communication, nursing service attitude, professional technology, nursing environment, knowledge propaganda, and education in the research group were significantly higher than those in the control group (*P* < 0.05) (see Table 4).

## 4. Discussion

Healthcare quality is not just the sum of a nurse's academic concepts, operating behaviors, operational levels, and healthcare impact, it is also the fundamental information of clinical governance. It is directly concerned with the safety and well-being of sick people. The patient care quality has a direct impact on the clinic's medical examination value [14]. Nursing quality management refers to the comprehensive management measures taken to reach the highest standard of nursing quality. At the same time, that is a significant managerial criterion for improving nursing knowledge and the appearance of nursing staff as well [15]. With the implementation of medical reform and the transformation of medical model, the requirements of general public and sick people for hospital nursing service quality are increasing day by day, which makes the management of nursing quality particularly important [16]. Studying how to improve nursing quality has evolved in the major objective of healthcare nurse staffing [17]. In recent years, both nursing theoretical research and clinical practice research have made some progress. More supervisors and hospital staff utilize new organizational strategies to healthcare quality control and effectively practice, so that the healthcare control model continues to improve and improve [18, 19], so that nurses are satisfied and the society can rest assured. Among them, the PDCA circuit method proved to be among the most strong and efficient frameworks for healthcare staff [20].

The PDCA cycle is a basic method of total quality management. The PDCA cycle is divided into four stages, namely, the planning phase (plan), the implementation phase (do), the inspection phase (check), and the processing phase (action). The four stages do not need to be completed successively but can be promoted at the same time. The result of a cycle can become the premise of a new cycle, so that all the problems are solved [21]. The specific application way of the PDCA cycle in practical work is to put forward problems and work objectives, analyze and find out the causes of the problems and current difficulties, work out corresponding solutions accordingly, ensure the effective implementation of the plan in a reasonable way, through timely evaluating the efficacy of implementations, modify goals and experience, and enter the new cycle with unsolved problems [22, 23], so that all kinds of work can be optimized. The PDCA cycle is a management mode that embodies the unified concept of combining practice with cognition, practice and cognition cycle. It is a powerful strategic tool that is always getting better and better [24]. Because the PDCA cycle itself is in line with the law and widely applicable [25], it was first valued and applied in enterprise management and has been verified by the actual effect [26]. The concept and logic of PDCA cycle are rigorous, the implementation level is three-dimensional and rich, and it has a broad application space in different fields. All industries regard it as an effective means to improve the management model and try to apply it in various management links [27–29]. Through the comparison of nursing quality in different wards, the different results were found: work enthusiasm was found in the work itself, workload, personal growth and development, work recognition, work management scores, and coworkers in the research group. The scores of relationships and family and work balance were greater than those of the control group. The nursing quality result suggested the nursing quality of gynecological operation area, emergency operation area, comprehensive operation area, and surgical operation area in research nurses was significantly better than the control cases (*P* < 0.05). The quality management of nursing documents showed that the number of problems in nursing documents such as nursing record displayed fewer than control group (*P* < 0.05). The personal quality-controlled checking in the medical department showed that the points of ward governance, head nurse management quality control examination, first-level nursing, recovery, publications on therapeutics, pill governance, and healthcare documentation in the research group were higher than control group (*P* < 0.05). The teamwork ability implied the scores of interpersonal communications, problem definition, project division, team evaluation assistance and motivation, data collection, interpretation, and extraction of results in the observation group were remarkably greater than those of control group (*P* < 0.05). The satisfaction mark showed that the scores of care information exchange, advanced technologies, attitude towards care providing, healthcare establishing, knowledge publicity, and learning in the researches were markedly more than those of the control group (*P* < 0.05). Therefore, through the analysis of the above results, we think that the PDCA cycle makes nursing quality monitoring more planned and systematic and promotes the improvement of nursing quality, thanks to its targeted, interlinked and layer-by-layer implementation. There are not only scientific practical investigation but also specific improvement measures, and through the follow-up implementation and effect evaluation of strengthening measures, the “soft index” of nursing management can be effectively transformed into “hard index.”

The concrete embodiment of the ability of teamwork is that under the guidance of the same goal, the participants strive to achieve the set goals by cooperating with each other and complementing each other, develop towards their own goals, and complete the task efficiently. Thus, it can be seen that the core of team cooperation ability is the balance between individual interests and overall interests, which forms the cohesion among the members, ensures the efficient operation of the team, promotes the common growth of the members, and finally completes the task [30]. And through performance evaluation, fully considering the difficulty and time-consuming work, while giving full play to the positive incentive role of bonuses, can effectively improve nurses' sense of achievement and satisfaction in work. Therefore, the analysis of the above differences may be related to the full play of nurses' own strengths under the PDCA cycle management mode and the full embodiment of the principle of “excellent work, excellent pay” and “more pay for more work.”

To sum up, compared with the traditional clinical nursing management, the application of the PDCA circulation management mode can effectively improve the quality of hospital nursing work, strengthen nurses' ability of teamwork, improve nurses' work efficiency and enthusiasm, enhance their sense of achievement and achievement in clinical nursing work, then improve patient satisfaction, and enhance the reputation and competitiveness of hospitals. Therefore, the PDCA management model is worth popularizing and applying in clinic.

## Figures and Tables

**Figure 1:** Comparison of nursing quality in each area of the two groups (*x̅*±*s*, points).

**Figure 2:** Comparison of the problems existing in the quality management of nursing documents between the two groups of nurses (*n*/%).

**Table 1:** Comparison of work enthusiasm between the two groups (*x̅*±*s*, points).

Group	*N*	Family/work balance	Work is recognized	Personal growth and development	Wages and benefits	The work itself	Relationship with colleagues	Workload	Manage
C group	80	6.12 ± 1.22	13.84 ± 2.93	14.59 ± 1.95	14.96 ± 3.11	17.92 ± 1.21	19.82 ± 1.35	24.96 ± 1.55	23.96 ± 3.91
R group	80	12.95 ± 2.41	18.49 ± 2.53	19.38 ± 3.35	19.86 ± 2.45	21.95 ± 3.13	23.69 ± 1.24	28.91 ± 2.14	30.95 ± 2.11
*t*		22.615	10.743	11.052	11.069	10.741	18.883	13.370	14.071
*P*		<0.01	<0.01	<0.01	<0.01	<0.01	<0.01	<0.01	<0.01

**Table 2:** Comparison of individual quality control scores between two groups of clinical departments (*x̅*±*s*, points).

Group	*N*	Ward management	Rescue and treatment of articles	Drug management	Special first-class nursing	Nursing documents	Head nurse management
C group	80	85.95 ± 2.11	86.93 ± 2.34	86.93 ± 2.45	86.92 ± 2.45	87.91 ± 2.67	85.93 ± 2.16
R group	80	94.82 ± 1.56	94.29 ± 2.15	95.85 ± 1.21	91.68 ± 2.33	96.81 ± 2.22	94.86 ± 2.11
*t*		30.233	20.715	29.197	12.592	22.925	26.451
*P*		<0.01	<0.01	<0.01	<0.01	<0.01	<0.01

**Table 3:** Comparison of team cooperation ability between the two groups of nurses (*x̅*±*s*, points).

Group	*N*	Interpersonal communication	Team evaluation	Team assistance	Team motivation	Problem definition	Project division of labor	Data collection	Interpretation of information	Extraction result
C group	80	5.95 ± 0.55	5.39 ± 1.21	6.05 ± 1.21	6.41 ± 1.21	5.92 ± 1.21	6.08 ± 1.21	5.89 ± 0.11	5.82 ± 0.42	6.12 ± 1.21
R group	80	7.28 ± 0.33	8.05 ± 0.31	7.83 ± 0.23	6.93 ± 1.33	7.06 ± 1.22	7.42 ± 0.53	7.58 ± 1.22	7.49 ± 1.28	8.05 ± 0.42
*t*		18.546	19.047	12.926	2.586	5.943	9.073	12.339	11.087	13.477
*P*		<0.01	<0.01	<0.01	<0.01	<0.01	<0.01	<0.01	<0.01	<0.01

**Table 4:** Comparison of patient satisfaction scores between the two groups (*x̅*±*s*, points).

Group	*N*	Nursing communication	Professional technology	Nursing service attitude	Nursing environment	Knowledge propaganda and education
C group	80	15.63 ± 1.95	14.96 ± 2.34	15.91 ± 2.94	18.84 ± 2.91	15.82 ± 1.95
R group	80	18.93 ± 1.58	18.49 ± 1.94	19.39 ± 1.41	25.91 ± 1.22	19.94 ± 0.52
*t*		11.760	10.387	9.546	20.040	18.259
*P*		<0.01	<0.01	<0.01	<0.01	<0.01

## Data Availability

No data were used to support this study.
